RETRACTED

# Analysis of Prognostic Factors and Treatment Modes of Patients with Recurrent Endometrial Carcinoma

**DOI:** 10.1155/2021/8793187

**Published:** 2021-10-18

**Authors:** Yi Li, Dong Yang, Shuangjian Yang

**Affiliations:** ^1^The First Affiliated Hospital, Department of Obstetrics and Gynecology, Hengyang Medical School, University of South China, Hengyang, Hunan 421001, China; ^2^The First Affiliated Hospital, Department of Radiation Oncology, Hengyang Medical School, University of South China, Hengyang, Hunan 421001, China

## Abstract

**Objective:**

Recurrence of endometrial cancer after initial treatment can be complex and difficult to treat. The current main treatment modalities for patients with recurrent endometrial cancer (REC) include chemotherapy, radiotherapy, and surgery, which vary according to the individual patient. However, REC is often associated with a poor prognosis, and it is therefore important to investigate the risk factors affecting REC prognosis and to explore appropriate treatment modalities to improve the prognosis and treatment strategies for patients with REC.

**Methods:**

Totally, 100 patients with REC admitted to our hospital from January 2013 to January 2018 were chosen to be research objects. Their pathological data were analyzed, including age, disease-free interval (DFI), recurrence site, and treatment plan after relapse (definitive local therapy (DLT) and palliative chemotherapy (PC)). According to these parameters, univariate and multivariate factors affecting the prognosis of REC patients and the curative effect of PC were analyzed, and the 3-year overall survival (OS) curve and progression-free survival (PFS) curve were drawn.

**Results:**

After 3 years of follow-up, 30 patients had a poor prognosis and 70 had a good prognosis, according to which a single multifactorial analysis was performed for different prognoses, where the results of the single-factor analysis showed significant differences between patients with different prognoses in terms of pathomorphology, pathological grading, TFI, and treatment modality after relapse. Further multifactorial analysis showed that TFI and treatment modality after recurrence were independent factors affecting poor prognosis in REC patients. The 3-year OS and 3-year PFS of REC patients were 74.00% and 70.00%, respectively. Patients whose DFI was less than 12 months or treated with PC after relapse were notably associated with lower levels of 3-year OS and 3-year PFS. In addition, radiotherapy and chemotherapy, DFI, and chemotherapy plan after primary surgery were independent risk factors that affected the PC efficacy of REC patients.

**Conclusion:**

DFI and treatment mode after relapse are independent factors affecting the prognosis of REC patients. DLT can obviously improve the prognosis of REC patients. For patients who can only choose PC, chemoradiotherapy and DFI after primary surgery are helpful to predict the chemotherapy effect, and the combination of paclitaxel and platinum drugs should be the first choice for chemotherapy.

RETRACTED

## 1. Introduction

Endometrial carcinoma (EC) is a group of epithelial malignant tumors occurring in the endometrium, with adenocarcinoma originating from the endometrial glands being the most common, and is one of the most common gynaecological malignancies, posing a serious threat to women's health [1, 2]. Although there are about 319,000 EC cases worldwide, the clinical symptoms of EC appear early, so that the vast majority of patients can be diagnosed before extrauterine metastasis of the tumor, and the diagnosis is mostly made at an early stage [3]. Most patients with EC have a good survival outcome after systemic therapy and their tumor recurrence rate is low, but once the tumor has recurred, the prognosis is often poor. Recurrent endometrial cancer (REC) is a great clinical challenge in the management of EC. Approximately 10–15% of patients with early-stage EC develop tumor recurrence after staged surgery, and among women with EC, there is a high incidence of tumor recurrence in the two to three years following systemic therapy [4–6]. Early EC can be screened out and cured at an early stage, but REC predicts poor prognosis [7]. Therefore, it is of great significance to study the prognostic factors and treatment modes of REC for improving the prognosis and treatment strategies of these patients.

The current treatment option for REC is mainly palliative chemotherapy (PC), which is of some significance for lesion control and survival extension, but some studies have found that systemic chemotherapy has significant toxic side effects and is difficult to achieve eradication, so patient survival time improvement is more limited under this treatment strategy [8]. Studies [9] have found that definitive local therapy (DLT) can also be used as a treatment scheme for REC patients, that is, removing local lesions through surgery and radiotherapy, so as to achieve the purpose of salvage therapy. However, there are few reports on this treatment mode in REC at present. Studies have reported that DLT is often used in recurrent or metastatic tumor diseases. DLT combined with lycopene has a high safety and stable effect in the treatment of recurrent prostate cancer. It is conducive to improving the overall survival (OS) of metastatic cervical cancer patients [10, 11]. Paclitaxel combined with platinum drugs is a common chemotherapy option for REC patients. As a remission induction therapy, it can improve the lifetime of patients [12, 13].

RETRACTED

This study included 100 patients with REC. It mainly analyzes the prognostic factors and treatment modes of patients, hoping to provide clinical reference for the treatment of patients.

## 2. Data and Methods

### 2.1. General Data

Totally, 100 patients with REC admitted to our hospital from January 2013 to January 2018 were selected as the research objects, with an average age of 64.25 ± 7.26 years. Information related to the patient's age, International Society of Obstetrics and Gynaecology staging, chemoradiotherapy after initial surgery, depth of invasive muscular invasion, type of pathology, grade of pathology, mode of treatment after recurrence, and site of recurrence was recorded. This study was approved by the Ethics Committee of our hospital, and all subjects had signed a fully informed consent form.

The inclusion criteria were as follows: patients diagnosed as EC by pathology [14] and had a recurrence after the initial treatment, expected survival period of patients was not less than 12 months, patients actively cooperated with 3-year follow-up, and patients met DLT or PC treatment conditions. All patients underwent full surgical-case staging. Clinical, pathological, and follow-up information was complete for all patients.

The exclusion criteria were as follows: patients complicated with malignant tumor, severe organ dysfunction, mental illness, communication disorder, or infectious diseases, patients had taken any drug with potential influence on the study indicators within the last six months, pregnant and lactating patients, and patients who had undergone secondary surgery or postoperative adjuvant treatment in our hospital after treatment in an external hospital.

### 2.2. Treatment Mode

DLT: it is a local salvage treatment for localized recurrent lesions (such as local pelvic recurrence and localized or isolated distant metastasis), with the purpose of achieving complete remission of the tumor again. Surgery and radiotherapy are main treatment methods in DLT. Systemic chemotherapy could be used as adjuvant therapy to consolidate the effect of surgery and radiotherapy.

PC: for patients who were not suitable for DLT, systemic chemotherapy was adopted, and the purpose of chemotherapy at this time was palliative.

### 2.3. Efficacy Evaluation

Efficacy evaluation was based on Response Evaluation Criteria in Solid Tumors (RECIST) version 1.1 [15], including complete response (CR), partial response (PR), stable disease (SD), and progressive disease (PD). The percentage of CR and PR in the total number of cases was the objective response rate (ORR).

RETRACTED

### 2.4. Follow-Up

The patients were followed up for 3 years from the end of the first treatment. Patients were followed up by telephone, and information on their survival was also obtained by combining relevant follow-up records from our follow-up department and return to hospital for review. The follow-up time was March, June, September, and December of each year.

### 2.5. Statistical Analysis

GraphPad Prism 6 (GraphPad Software, San Diego, USA) was used for data analysis and picture generation. The counting data were expressed by the number of cases/percentage (*n*, %), and the comparison of the counting data between groups was performed by the chi-square test. When the theoretical frequency in the chi-square test was less than 5, the continuity correction chi-square test was adopted. The measurement data were expressed by mean ± standard deviation (mean ± SD). The independent sample *t*-test was utilized for comparison of measurement data between groups. Univariate and multivariate Cox regression analysis was applied to analyze the independent prognosis or risk factors affecting the prognosis of REC patients and PC efficacy. The Kaplan–Meier method was utilized to draw the 3-year OS and progression-free survival (PFS) curves of REC patients. The log-rank test was used for comparison. When *P* < 0.05, the difference was statistically significant.

## 3. Results

### 3.1. Clinicopathological Data of REC Patients

In this study, the average age of REC patients was 64.25 ± 7.26 years, showing mainly FIGO stage of I/II stage (85.00%), chemoradiotherapy after primary surgery of 74 cases (74.00%), main infiltrating muscularis of ≥1/2 (56.00%), main pathological pattern of endometrioid adenocarcinoma (78.00%), main pathological grade of *G*3 (50.00%), main recurrent site of outside the pelvic cavity (60.00%), and main treatment mode after recurrence of DLT (41.00%) and PC (59.00%), as shown in Table 1.

### 3.2. Univariate and Multivariate Analysis on Prognosis of REC Patients

The 3-year follow-up was successfully completed. Patients with tumor progression or death were considered as the poor prognosis group (*n* = 30), and the rest were considered as the good prognosis group (*n* = 70). By comparing the difference of clinical parameters and related indexes between patients with poor prognosis and good prognosis, we found that there was no remarkable difference between the two groups in age, average age, FIGO stage, radiotherapy and chemotherapy after primary surgery, infiltrating muscularis, recurrence site, etc. (*P* > 0.05), while there was statistical difference in pathological pattern, pathological grade, DFI, and treatment mode after recurrence (*P* < 0.05). Multivariate Cox regression analysis was carried out for the different factors, and the results showed that DFI and treatment mode after relapse were independent prognostic factors affecting poor prognosis of REC patients (*P* < 0.05). REC patients whose DFI was less than 12 months and received treatment of PC after relapse had increased risk of poor prognosis, as shown in Tables 2–4.

RETRACTED

### 3.3. OS and PFS Curves of REC Patients

We plotted the 3-year OS and 3-year PFS curves of patients under the influence of DFI or treatment mode after relapse based on the above results. It can be seen that the 3-year OS was 74.00% (74/100) and 3-year PFS was 70.00% (70/100). Patients with DFI less than 12 months had notably lower levels of 3-year OS and 3-year PFS, while patients undergoing PC treatment mode after relapse had remarkably lower levels of 3-year OS and 3-year PFS, as shown in Figure 1.

### 3.4. Analysis of Factors Affecting PC Efficacy of REC Patients

In this study, there were 59 patients who received PC. Among them, those with CR and PR were enrolled in the effective group (*n* = 27), and the rest were enrolled in the ineffective group (*n* = 32), with an ORR of 45.76% (27/59). The difference of clinical parameters and related indexes between the effective group and ineffective group was compared. There was no remarkable difference between the two groups in age, average age, FIGO stage, infiltrating muscularis, pathological pattern, pathological grade, relapse site, paclitaxel + platinum drug regimen, etc. (*P* > 0.05), while there was statistical difference in radiotherapy and chemotherapy, DFI, and chemotherapy regimen after primary surgery (*P* < 0.05). Multivariate Cox regression analysis was carried out on the factors with differences. The results showed that radiotherapy and chemotherapy, DFI, and chemotherapy regimen after primary surgery were independent risk factors affecting the PC efficacy of REC patients (*P* < 0.05). The risk of PC treatment failure increased for REC patients with radiotherapy and chemotherapy, DFI < 12 months, and other treatment schemes after primary surgery, as shown in Tables 5–7.

## 4. Discussion

EC is a common gynaecological tumor, and its incidence is on the rise. REC is defined as EC in complete remission after systemic treatment, followed by the appearance of a new lesion of the same pathological histological type as the primary tumor some time later. REC is the leading cause of death from gynaecological cancers in women due to its high recurrence rate, and treatment of recurrence depends on the specific site of recurrence, the oncological nature of the lesion, the disease-free interval, the patient's overall health status, and the availability of postoperative adjuvant therapy [16–18].Therefore, it may be of great value to study the prognostic factors and treatment modes of REC for improving the survival of patients.

RETRACTED

In this study, the average age of REC patients was 64.25 ± 7.26 years, mainly showing FIGO stage I/II (85.00%), invasive myometrium ≥1/2 (56.00%), and pathological grade G3 (50.00%). Takahashi et al. [19] pointed out that the risk factors for the occurrence of stage I-II REC include advanced age (≥60 years), higher pathological tumor grade, and muscular infiltration, which partially explains the rationality of the main manifestations of this REC cohort, such as higher average age, infiltrating myometrial ≥1/2, pathological grade *G*3, etc. Although patients in stage I-II often have good prognosis, they still have different degrees of recurrence risk [20]. In addition, deep infiltrating muscularis and high pathological grade are important prognostic factors for REC patients, which are related to the increase and metastasis of tumor vascular infiltration [21].

Further analysis showed that DFI and treatment mode after relapse were independent prognostic factors affecting poor prognosis of REC patients, and the risk of poor prognosis of REC patients with DFI less than 12 months and PC after relapse was increased. The DFI is the disease-free interval and is an important prognostic indicator for patients with stage I–IV REC. DFI less than 12 months often symbolizes short-term recurrence, which we speculate may be related to poor treatment [22, 23]. In the study of Murakawa et al. [24], the treatment mode is obviously related to OS of tumor patients, which is different from our research results. As for the relationship between PC and poor prognosis of REC patients, we speculate that this may be related to the nonlocality of the lesion range. We also plotted the survival curves of 3-year OS and 3-year PFS affecting REC patients with DFI and treatment mode after relapse. The results showed that DFI less than 12 months and PC as treatment after relapse were remarkably correlated with 3-year OS and 3-year PFS, suggesting that DFI or treatment mode after relapse may be used as prognostic factors for REC patients, and REC patients adapted DLT treatment scheme were more likely to have higher 3-year OS. In addition, in this study, the 3-year OS and 3-year PFS of REC patients were 74.00% and 70.00%, respectively, which is similar to the research results of Lan et al. [25]. Finally, we also analyzed the independent risk factors that affected the PC efficacy of REC patients. The results showed that radiotherapy and chemotherapy after primary surgery, DFI, and chemotherapy plan were independent factors in this aspect. The risk of PC failure for REC patients receiving radiotherapy and chemotherapy, DFI less than 12 months after primary surgery, and other treatment plans increased. Similar to ours, the team of Shimamoto pointed out that the effect of chemotherapy on the therapeutic effect of REC patients may be determined by DFI, and patients with DFI ≥12 months have better therapeutic response [23]. For patients who received radiotherapy and chemotherapy after primary surgery, we speculated that the body might already have certain drug resistance, which more or less affected the effectiveness of the treatment mode after relapse. Studies have reported that the therapeutic effectiveness of paclitaxel combined with platinum drugs chemotherapy in REC patients has been confirmed. Compared with platinum drugs alone, the combined scheme is more conducive to improving patients' 5-year PFS, which reflects the reliability of the combined scheme [26].

RETRACTED

Although DFI and treatment mode are found to be independent factors affecting the prognosis of REC patients and the efficacy of PC, there is still room for improvement in this study. First of all, we can supplement the research on the basic mechanism of REC occurrence and explore the underlying principle from the molecular level. In addition, we can further expand the study of treatment modes, such as molecular targeted therapy, which may help to further optimize the treatment mode for improving the prognosis of REC patients. We will gradually improve our research around the above two aspects in the future.

To sum up, DFI and treatment mode of REC patients are independent factors affecting the prognosis. Active use of DLT is helpful to improve the prognosis of patients. For patients who can only use PC, DFI and radiotherapy and chemotherapy after primary surgery are important indicators for predicting the curative effect, and paclitaxel combined with platinum chemotherapy can be the first choice.

## Figures and Tables

**Figure 1:** OS and PFS curves of REC patients. (a, b) 3-year OS curve and (c, d) 3-year PFS curve of patients affected by DFI or treatment mode after relapse.

**Table 1:** Clinicopathological data of REC patients (*n* (%) and mean ± SD).

Factors	Patients (*n* = 100)
*Age (years)*	
<65	55 (55.00)
≥65	45 (45.00)

Average age (years)	64.25 ± 7.26

*FIGO stage*	
I	68 (68.00)
II	17 (17.00)
III	10 (10.00)
IV	5 (5.00)

*Radiotherapy and chemotherapy after primary surgery*	
No	26 (26.00)
Yes	74 (74.00)

*Infiltrating muscularis*	
Without	20 (20.00)
<1/2	24 (24.00)
≥1/2	56 (56.00)

*Pathological pattern*	
Endometrioid adenocarcinoma	78 (78.00)
Serous adenocarcinoma	22 (22.00)

*Pathological grade*	
*G*1	28 (28.00)
*G*2	22 (22.00)
*G*3	50 (50.00)

*DFI (months)*	
<12	48 (48.00)
≥12	52 (52.00)

*Recurrence site*	
Pelvic cavity	40 (40.00)
Outside the pelvic cavity	60 (60.00)

*Treatment mode after relapse*	
DLT	41 (41.00)
PC	59 (59.00)

RETRACTED

**Table 2:** Univariate analysis on prognosis of REC patients (*n* (%) and mean ± SD).

Factors	*n*	Good prognosis (*n* = 70)	Poor prognosis (*n* = 30)	*χ* ^2^/*t*	*P*
*Age (years)*				0.433	0.511
<65	55	40 (57.14)	15 (50.00)		
≥65	45	30 (42.86)	15 (50.00)		

Average age (years)	100	63.02 ± 6.18	65.03 ± 5.36	1.548	0.125

*FIGO stage*				5.630	0.131
I	68	52 (74.29)	16 (53.33)		
II	17	11 (15.71)	6 (20.00)		
III	10	5 (7.14)	5 (16.67)		
IV	5	2 (2.86)	3 (10.00)		

*Radiotherapy and chemotherapy after primary surgery*				1.198	0.274
No	26	16 (22.86)	10 (33.33)		
Yes	74	54 (77.14)	20 (66.67)		

*Infiltrating muscularis*				1.293	0.524
Without	20	12 (17.14)	8 (26.67)		
<1/2	24	18 (25.71)	6 (20.00)		
≥1/2	56	40 (57.15)	16 (53.33)		

*Pathological pattern*				5.372	0.021
Endometrioid adenocarcinoma	78	59 (84.29)	19 (63.33)		
Serous adenocarcinoma	22	11 (15.71)	11 (36.67)		

*Pathological grade*				12.518	0.002
*G*1	28	25 (35.71)	3 (10.00)		
*G*2	22	18 (25.71)	4 (13.33)		
*G*3	50	27 (38.58)	23 (76.67)		

*DFI (months)*				11.020	<0.001
<12	48	26 (37.14)	22 (73.33)		
≥12	52	44 (62.86)	8 (26.67)		

*Recurrence site*				1.786	0.181
Pelvic cavity	40	31 (44.29)	9 (30.00)		
Outside pelvic cavity	60	39 (55.71)	21 (70.00)		

*Treatment mode after relapse*				5.530	0.019
DLT	41	34 (48.57)	7 (23.33)		
PC	59	36 (51.43)	23 (76.67)		

**Table 3:** Cox multivariate regression analysis assignment.

Factors	Variable	Assignment
Pathological pattern	*X*1	Endometrioid adenocarcinoma = 0, serous adenocarcinoma = 1
Pathological grade	*X*2	*G*1 = 0, *G*2 = 1, *G*3 = 2
DFI	*X*3	≥12 = 0, <12 = 1
Treatment mode after relapse	*X*4	DLT = 0, PC = 1

**Table 4:** Multivariate analysis on prognosis of REC patients.

Factor	*β*	S.E	Wald	*P*	OR	95% CI
Pathological pattern	0.441	0.284	3.001	0.211	1.554	0.891–2.712
Pathological grade	0.545	0.289	3.143	0.095	1.724	0.979–3.039
DFI	0.824	0.375	4.816	0.030	2.280	1.093–4.754
Treatment mode after relapse	1.263	0.539	5.415	0.018	3.536	1.339–10.170

**Table 5:** Univariate analysis of PC effect on REC patients (*n* (%) and mean ± SD).

Factors	*n*	Effective (*n* = 27)	Ineffective (*n* = 32)	*χ* ^2^/*t*	*P*
*Age (years)*				0.273	0.601
<65	35	17 (62.96)	18 (56.25)		
≥65	24	10 (37.04)	14 (43.75)		

Average age (years)	59	63.78 ± 5.30	65.02 ± 5.68	0.861	0.393

*FIGO stage*				1.076	0.783
I	35	15 (55.56)	20 (62.50)		
II	12	7 (25.93)	5 (15.63)		
III	9	4 (14.81)	5 (15.63)		
IV	3	1 (3.70)	2 (6.24)		

*Radiotherapy and chemotherapy after primary surgery*				7.367	0.007
No	28	18 (66.67)	10 (31.25)		
Yes	31	9 (33.33)	22 (68.75)		

*Infiltrating muscularis*				2.255	0.324
Without	11	6 (22.22)	5 (15.63)		
<1/2	14	4 (14.81)	10 (31.25)		
≥1/2	34	17 (62.97)	17 (53.12)		

*Pathological pattern*				2.186	0.139
Endometrioid adenocarcinoma	45	23 (85.19)	22 (68.75)		
Serous adenocarcinoma	14	4 (14.81)	10 (31.25)		

*Pathological grade*				3.688	0.158
*G*1	15	10 (37.04)	5 (15.63)		
*G*2	14	6 (22.22)	8 (25.00)		
*G*3	30	11 (40.74)	19 (76.67)		

*DFI (months)*				16.076	<0.001
<12	32	7 (25.93)	25 (78.13)		
≥12	27	20 (74.07)	7 (21.87)		

*Recurrence site*				3.543	0.060
Pelvic cavity	25	15 (55.56)	10 (31.25)		
Outside pelvic cavity	34	12 (44.44)	22 (68.75)		

*Chemotherapy regimen*				14.019	<0.001
Paclitaxel + platinum drugs	40	25 (92.59)	15 (46.88)		
Others	19	2 (7.41)	17 (53.12)		

*Paclitaxel* *+* *platinum drug scheme*				0.293	0.589
Paclitaxel + cisplatin	24	12 (44.44)	12 (37.50)		
Paclitaxel + other platinum drugs	35	15 (55.56)	20 (62.50)		

RETRACTED

**Table 6:** Cox multivariate regression analysis assignment.

Factors	Variable	Assignment
Radiotherapy and chemotherapy after primary surgery	*X*1	No = 0, yes = 1
DFI	*X*2	≥12 = 0, <12 = 1
Chemotherapy regimen	*X*3	Paclitaxel + platinum drugs = 0, others = 1

**Table 7:** Multivariate analysis on PC efficacy of REC patients.

Factor	*β*	S.E	Wald	*P*	OR	95% CI
Radiotherapy and chemotherapy after primary surgery	0.831	0.353	9.882	0.001	2.296	1.149–4.585
DFI	0.728	0.346	6.552	0.001	2.071	1.051–4.080
Chemotherapy regimen	0.957	0.340	12.233	<0.001	2.604	1.337–5.070

## Data Availability

The data used during the current study are available from the corresponding author.
